# Comparison of a Small Dose of Oxycodone and Sufentanil for the Prevention of Sufentanil-Induced Cough during General Anesthesia Induction: A Prospective Randomized Controlled Trial

**DOI:** 10.1155/2022/7924643

**Published:** 2022-06-17

**Authors:** Lingli Shi, Lu Liu, Yong He, Yuling Yang, Huanhuan Ni

**Affiliations:** ^1^Department of Anesthesiology, Children's Hospital of Nanjing Medical University, Nanjing 210017, China; ^2^Department of Anesthesiology, The Second Affiliated Hospital of Nanjing Medical University, Nanjing 210003, China

## Abstract

**Background:**

Sufentanil is widely used during anesthesia induction. However, it can cause coughing via different mechanisms. This study is aimed at evaluating the effectiveness of a small dose of oxycodone and sufentanil in suppressing sufentanil-induced cough (SIC) during general anesthesia induction.

**Methods:**

Of the 174 patients scheduled for elective surgery, 144 were eligible and randomly divided into 3 groups (*n* = 48). Five minutes before sufentanil bolus (0.4 *μ*g/kg), patients in group O received 0.02  mg/kg oxycodone intravenously within 5 s, those in group S received 0.02 *μ*g/kg sufentanil within 5 s, and those in group N received an equal volume of 0.9% normal saline within 5 s. Sufentanil was diluted to 5 *μ*g/ml and administered within 5  s after pretreatment. The incidence and severity of cough in the three groups were evaluated within 1 minute after sufentanil injection during the anesthesia induction. Their mean arterial pressure (MAP) and heart rate (HR) were recorded at T0 (after entering the operation), T1 (3 minutes after pretreatment), T2 (before intubation), and T3 (1 minute after intubation).

**Results:**

The incidences of cough in group N, group O, and group S were 20 (41.6%), 7 (14.5%), and 6 (12.5%), respectively. Compared with group N, patients from group O and group S exhibited significantly reduced incidence and severity of cough, and the severity of cough in group O and group S was significantly reduced compared with group N (*P* < 0.05). No significant differences in the rangeability of MAP and HR were noted at the four time points in the three groups (*P* > 0.05)*. Conclusion*. Preconditioning using intravenous oxycodone (0.02 mg/kg) or sufentanil (0.02 *μ*g/kg) could represent an effective approach to reducing SIC in anesthesia induction and was associated with relatively stable hemodynamic state during general anesthesia. This trial is registered at Chinese Clinical Trial Registry with registration number ChiCTR1900021087.

## 1. Background

Sufentanil has some advantages, such as a fast onset time, strength of analgesic function, and cardiovascular stability, and is considered an ideal option that is widely used by anesthesiologists for general anesthesia [1]. However, sufentanil can cause coughing during general anesthesia induction. The incidence of sufentanil-induced cough (SIC) during anesthesia has been reported by different studies to range from 16 to 47% [2–4].

Although SIC appears to be transient in most cases, this pathological condition may result in disastrous consequences in patients with compromised central nervous system (CNS) injury, open eye injury, or cardiovascular diseases. Thus, certain patients should be maintained on an absolutely stable hemodynamic status and intracranial or intraocular pressure during anesthesia induction. Explosive coughs may increase intra-abdominal pressure, increasing the risk of regurgitation and aspiration [5]. Clinical interventions, such as pretreatment with drugs (butorphanol, dezocine, remifentanil, and dexmedetomidine), changing the administration route or diluting the concentration of sufentanil, have been reported to reduce SIC [1–3, 6–13]. However, the interventions could not be widely implemented in clinical practice due to several side effects such as long onset time, bradycardia, and respiratory depression. Thus, identifying alternative drugs to overcome SIC is urgently needed.

Oxycodone is a derivative of thebaine and is mainly used to alleviate perioperative pain. It can inhibit *μ* and *κ* agonists and exert obvious antitussive effects by directly acting on the cough center of the medulla oblongata [14]. A previous study found that preemptive use of a small dose of opioids could suppress opioid-induced cough without applying additional drugs [10, 15, 16]. In this study, we explored the effect of pretreating patients with a small dose of oxycodone and sufentanil on the incidence and severity of SIC when larger doses of sufentanil (0.4 *μ*g/kg) were subsequently administered during the induction of general anesthesia.

## 2. Methods

This study was approved by the institutional ethics committee of the Second Affiliated Hospital of Nanjing Medical University and registered at the Chinese Clinical Trial Registry with registration number ChiCTR1900021087. All participants provided written informed consent. In addition, this study adhered to the CONSORT guidelines.

### 2.1. Participants

A total of 174 patients with ASA physical status I-II, aged 18–65 years, and BMI 18.5–30 kg/m^2^ and scheduled for elective surgery under general anesthesia between April 2018 and March 2019 were enrolled in this study. The exclusion criteria included a history of asthma or chronic obstructive pulmonary disease (COPD); upper respiratory tract infection in the last two weeks; smoking, bronchodilator, or steroid therapy; chronic administration of opioids; impaired kidney and liver function; and allergy to oxycodone, anticough medication, or angiotensin-converting enzyme (ACE) inhibitors. Patients were also excluded if they were diagnosed with increasing intracranial or intraocular pressure.

### 2.2. Study Protocol

The scheduled patients were randomly divided into three groups (*n* = 48), namely, groups O, S, and N, using computer-generated random numbers. No pretreatment drug was administered before surgery. Upon entering the operating room, the patients' heart rate, invasive arterial blood pressure, respiratory rate, and oxygen saturation were monitored. Venous access was established on the wrist cephalic vein of the nondominant hand with a 20-G intravenous cannula, and an IV cannula was connected to T-connectors for drug infusion and injection. Intravenous perfusion was given using the Ringers' solution at 8 ml/kg/h after venous catheterization. The vertical distance from the drip bottle to the venous access was kept at 70 cm in all the patients in this study. Patients were given 100% oxygen by a face mask.

Group O patients were administered 0.02 mg/kg oxycodone (diluted to 2 ml) intravenously within 5 s, group S patients were administered 0.02 mg/kg sufentanil (diluted to 2 ml) intravenously within 5 s, and group N patients were administered 2 ml of normal saline. The preparation and administration of the pretreated drugs were performed by nurse anesthetists and anesthesiologists, respectively. Five minutes after pretreatment with the drugs, 0.4 *μ*g/kg sufentanil with an injection time of 5 s was administered to all patients. A stopwatch was used to monitor the time. After sufentanil injection, the symptoms of the explosive cough, including the number and severity, were recorded within 1 min by an anesthetist nurse who was blinded to the study. Depending on the number of coughs within 1 min, the patient was classified into four grades: 0 (no cough), 1 (mild, 1-2 times), 2 (moderate, 3–5 times), and 3 (severe, >5 times). Anesthesia induction was subsequently completed with 2 mg/kg propofol and 0.6 mg/kg rocuronium, and orotracheal intubation was performed 5 minutes later.

MAP and HR were recorded at baseline after entering the operation (T0), 3 min after injecting the pretreatment (T1), before orotracheal intubation (T2), and 1 min after orotracheal intubation (T3). We excluded patients who had unacceptable hypertension (≥160/90 mmHg) for the three measurements after calming down for 5 min.

### 2.3. Sample Size Determination

Sample size estimates were performed using the PASS 11 software (PASS, Kaysville, UT, USA). According to our pilot study, the incidence of cough induced by 0.4 *μ*g/kg sufentanil was 40% (8/20). The incidence was reduced to 15% (3/20) after pretreatment with 0.02 mg/kg oxycodone, and pretreatment with a dose of 0.02 *μ*g/kg sufentanil reduced the incidence of SIC to 18% (4/22). To achieve 80% statistical power with *α* = 0.05, each group would require no less than 46 patients. Considering the 20% drop-out rate, we recruited 58 patients in each group.

### 2.4. Statistical Analysis

The SPSS 22.0 software (IBM Corp, Armonk, NY, USA) was used for statistical analysis. Data are expressed as the mean ± standard deviation for continuous variables or *n* patients (%). Repeated measure ANOVA was applied to analyze the quantitative variables in three groups for MAP and HR at different time points. The incidence of cough (categorical data) was compared with the chi-squared test, and Bonferroni's correction was used for pairwise comparisons. The grade data for cough severity were analyzed using the rank-sum test. *P* < 0.05 was considered statistically significant.

## 3. Results

### 3.1. Demographic Characteristics

In total, 174 patients were screened. Among them, 18 patients did not meet the inclusion criteria, 6 patients refused to participate, and 7 patients were excluded because of unacceptable hypertension. Finally, 144 patients participated in this study (Figure 1). Their demographic data (age, sex, BMI, and weight) and ASA physical status were not significantly different among the three groups (*P* > 0.05, Table 1).

### 3.2. Incidence and Severity of Cough for SIC

The incidences of cough in group N, group O, and group S were 20 (43.5%), 7 (14.5%), and 6 (12.2%), respectively. Compared with group N, group O and group S exhibited significantly reduced incidences of cough (*P* < 0.05, Table 2). No significant differences in incidences of cough between group O and group S were observed (*P* > 0.05). The severity of cough in group O and group S was significantly reduced compared with group N (*P* < 0.05), especially moderate and severe coughs. No significant differences were observed between group S and group N (*P* > 0.05, Table 2).

### 3.3. Hemodynamic Changes

No significant differences in the rangeability of MAP and HR were noted at the four indicated time points (T0 to T3) in the three groups (*P* > 0.05, Table 3).

## 4. Discussion

This study demonstrated that 0.02 mg/kg oxycodone and 0.02 *μ*g/kg sufentanil could effectively reduce the incidence and severity of SIC without aggravating hemodynamic changes.

Opioid analgesics are widely used in anesthesia induction and commonly possess the characteristics of strong analgesic effects and have slight impacts on hemodynamics. Cough is one of the side effects of intravenous sufentanil, and discrepancies in the incidence and severity of cough may depend on the injection dose, speed, and type of venous catheter. According to previous studies, the incidence of SIC varies between 16% and 47% [2–4]. Some specific patient groups, such as those with hypertension and intracranial or intraocular pressure increases, require stable anesthesia induction, and the occurrence of SIC could affect their surgery.

The mechanism of cough induced by opioids remains unclear; however, various studies have presented possibly reasonable explanations. It was reported that opioids could induce cough and reflex bronchoconstriction by inhibiting the central sympathetic nerves and activating the vagus nerve [17]. Pulmonary chemoreflex mediated by either irritant receptors or vagal C-fiber receptors adjacent to pulmonary vessels may represent another mechanism [17–19]. Opioid receptors exist in the tracheobronchial, and when they are irritated by opioids, the tracheal smooth muscles are stimulated and constrict [20]. Sufentanil-induced histamine release from lung mast cells [19] or supraglottic obstruction by soft tissue [21, 22] represents other likely mechanisms of cough. A study demonstrated that the closure of the vocal cord after injecting sufentanil might also be a major mechanism of cough [23].

Various pretreatment drugs, such as dexmedetomidine, ketorolac tromethamine, and lidocaine, that are used to suppress opioid-induced cough have been proven to be effective. However, potential risks and additional side effects have limited their clinical application. Zhou et al. [24] demonstrated that pretreatment with 0.6 *μ*g/kg dexmedetomidine infused intravenously over 10 mins could significantly decrease the incidence and severity of fentanyl-induced cough. However, anesthesia induction may require a prolonged infusion, and dexmedetomidine may cause bradycardia (<50 beats/min), respiratory depression, and hypotension. Tian et al. [2] found that applying ketorolac tromethamine 0.5 mg/kg intravenously before injecting 0.5 *μ*g/kg sufentanil could effectively reduce SIC. Ketorolac tromethamine is a nonsteroidal anti-inflammatory drug (NSAID) but may increase bleeding risks by inhibiting platelet function in the perioperative period. Relevant studies on ketorolac tromethamine suppressing SIC are lacking, and the prophylactic administration of ketorolac tromethamine (0.5 mg/kg) may not be the most appropriate dose for inhibiting SIC. In addition, 0.5 mg/kg lidocaine can effectively suppress remifentanil-induced cough when administered intravenously 1 min prior to remifentanil; however, lidocaine has a potential defect in systemic toxicity [25].

The onset time of intravenous oxycodone is 2-3 min, with a peak time of 5 min. Oxycodone is the only opioid double-receptor agonist available clinically, and the pharmacological effects include analgesia, antianxiety, and antitussive. According to previous studies, two possible mechanisms could potentially explain how oxycodone suppresses SIC. First, oxycodone may directly restrain the cough center in the medulla oblongata and then produce antitussive effects. Additionally, it may act on the *μ* and *κ* receptors of tracheal and bronchial trees to inhibit the reflex contraction of the trachea. There are a few studies associated with oxycodone inhibiting opioid-induced cough, and the proper antitussive dosage remains controversial. Dai et al. [14] concluded that 0.075 mg/kg oxycodone could prevent SIC effectively in general anesthesia induction and that the effect of suppression was dose-dependent. However, another study found that 0.025, 0.050, and 0.075 mg/kg of oxycodone could reduce the incidence and severity of SIC [26]. However, there was no difference among the groups, suggesting that intravenous injection of oxycodone could inhibit FIC in a dose-dependent manner. The conclusions remain different between the two studies, but the underlying mechanisms and cause urge further evaluation. Side effects may occur as the dosage increases; in particular, the risk of respiratory depression was higher when the dosage of oxycodone was increased to 0.1 mg/kg.

In this study, we established group S (0.02 *μ*g/kg sufentanil) based on several studies that reported pretreatment with a small dose of opioids could reduce opioid-induced cough. We chose a dosage of 0.02 *μ*g/kg, which depended on the equivalent dose conversion (sufentanil : oxycodone = 1000 : 1). Opioids may suppress the reflex of cough by directly affecting the cough center in the medulla, in which the preemptive dose used was less than required for analgesia. Hung et al. [16] showed that pretreatment with 25 *μ*g fentanyl could reduce the coughs caused by an induction dose of 125 *μ*g or 150 *μ*g of fentanyl. Pretreatment with 0.3 *μ*g/kg of remifentanil intravenously one minute before the analgesia of sufentanil could also effectively inhibit coughing caused by sufentanil [5]. One mechanism by which pretreatment inhibits opioid-induced cough may involve decreasing plasma concentration fluctuations. In addition, the preemptive use of opioids may deplete neurotransmitters in nerve fibers.

This study demonstrated that a small dose of 0.02 mg/kg oxycodone and 0.02 *μ*g/kg sufentanil could effectively reduce the incidence and severity of SIC. The mechanism of the two pretreatments that suppress cough remains to be elucidated. No adverse events, such as vomiting, hypotension, respiratory depression, and bradycardia, occurred when the small dosage was administered. The rangeability of MAP and HR remained synchronous at the four indicated time points, which might be due to the very low dose.

There were some limitations in this study. Few studies have shown the exact doses of pretreated sufentanil that could be used to suppress cough induced by sufentanil. The low dosage of sufentanil, which is used to suppress cough in this study, was obtained by referring to the equivalent doses of oxycodone. Additionally, in terms of applying a small equivalent analgesic dosage between oxycodone and sufentanil, there were no differences in inhibiting SIC. We do not know whether oxycodone could have a more effective antitussive function than sufentanil when increasing the dose of oxycodone to 0.03, 0.04, and 0.05 mg/kg.

## 5. Conclusion

Preconditioning using intravenous administration of a small dose of 0.02 mg/kg oxycodone and 0.02 *μ*g/kg sufentanil before general anesthesia could effectively reduce the incidence and severity of cough induced by sufentanil without adverse reactions during anesthesia induction.

## Figures and Tables

**Figure 1:** Flow diagram of the study.

**Table 1:** Demographic characteristics of patients in the three groups.

Characteristics	Group			*P* value		
	N	O^∗^	S^∗^	N vs. O	N vs. S	O vs. S
Age (years)	47.3 ± 11.8	45.6 ± 12.9	43.4 ± 11.9	0.7743	0.2643	0.6521
Gender (males/females)	15/33	17/31	15/33	0.9027	>0.9999	0.9027
Weight (kg)	62.4 ± 9.4	64.9 ± 10.1	64.3 ± 12.3	0.5833	0.7669	0.9898
BMI (kg/cm^2^)	23.6 ± 3.6	24.0 ± 3.1	23.9 ± 3.2	0.8243	0.8969	0.9880
ASA (I/II)	23/26	20/28	21/27	0.8146	0.9128	0.9774

Values are expressed as the mean ± standard deviation or as the number of cases.

**Table 2:** Incidence and severity of sufentanil-induced cough.

Cough	Group			*P* value		
	*N*	O^∗^	S	N vs. O	N vs. S	O vs. S
Incidence	20 (41.7)	7 (14.6)	6 (12.5)	0.0036	0.0015	0.9653
Severity						
0 (no cough)	28 (58.3)	41 (85.4)	42 (87.5)	0.0036	0.0015	0.9653
1 (mild)	8 (16.7)	4 (8.3)	5 (10.4)	0.4204	0.6130	0.9468
2 (moderate)	7 (14.6)	3 (6.3)	1 (2.1)	0.3029	0.1568	0.9272
3 (severe)	5 (10.4)	0 (0)	0 (0)	0.0133	0.0133	>0.9999

Note: values are numbers (percentage). ^∗^*P* < 0.05 vs. group N.

**Table 3:** Changes in MAP and HR in the three groups.

Variables	T0	T1	T2	T3	*P*
MAP (mmHg)					0.313
Group N	92.6 ± 13.8	91.0 ± 12.2	67.3 ± 13.8	86.9 ± 18.7	
Group O	90.3 ± 12.9	89.3 ± 13.7	64.6 ± 10.9	80.7 ± 13.9	
Group S	92.5 ± 11.5	92.2 ± 15.0	67.8 ± 8.4	82.4 ± 14.3	
HR (bpm)					0.335
Group N	76.7 ± 12.2	76.2 ± 10.7	66.8 ± 10.0	84.2 ± 14.5	
Group O	75.5 ± 9.0	74.5 ± 9.3	67.3 ± 11.3	85.2 ± 11.1	
Group S	80.0 ± 14.9	78.3 ± 12.9	70.6 ± 12.7	85.5 ± 11.4	

Values are expressed as the mean ± standard deviation. MAP: mean arterial pressure; HR: heart rate. T0 (after entering the operation), T1 (1 minute after the pretreatment), T2 (before intubation), and T3 (1 minute after intubation).

## Data Availability

The data used to support the findings of this study are available from the corresponding author upon request.

## Abbreviations

SIC: Sufentanil-induced cough
MAP: Mean arterial pressure
HR: Heart rate
CNS: Central nervous system
COPD: Chronic obstructive pulmonary disease
ACE: Angiotensin-converting enzyme.
